The article "Effect of Ejiao (Asini Corii Colla) and Turtle Carapace Glue on Gut Microbiota in Nude Mice with Uterine Fibroids Based on High-Throughput Sequencing of 16SrRNA Gene" was published in 2022. Journal: Evid Based Complement Alternat Med.

# Effect of Ejiao (Asini Corii Colla) and Turtle Carapace Glue on Gut Microbiota in Nude Mice with Uterine Fibroids Based on High-Throughput Sequencing of 16SrRNA Gene

**DOI:** 10.1155/2022/3934877

**Published:** 2022-07-06

**Authors:** Jia-Rou Qiu, Ming-Yao Yang, Ye-Lin Ma, Min-Chun Yang

**Affiliations:** ^1^Zhejiang Chinese Medical University, Hangzhou 310053, Zhejiang, China; ^2^Zhejiang Hospital, Hangzhou 310013, Zhejiang, China

## Abstract

**Objective:**

To observe the effects of Asini Corii Colla, turtle carapace glue, and other drugs on the intestinal flora of nude mice with uterine fibroids model, so as to provide evidence for the clinical application of drugs.

**Methods:**

Set up five groups: blank control group, turtle carapace glue group, turtle carapace glue and ejiao 4 : 1 mixed group, turtle carapace glue and ejiao 1 : 1 mixed group, and turtle shell glue and *Salvia miltiorrhiza* (danshen) 1 : 1 mixed group. Then, the model nude mice were fed ejiao, turtle carapace glue, and other corresponding drugs. Before administration, 2 weeks after administration, and 4 weeks after administration, the feces of the model nude mice were taken respectively, subpacked into labeled cryotubes, and stored at −80°C. All samples were sent for gene sequencing after completion. The differences in gut microbiota and abundance in different groups were compared by 16SrRNA segment sequencing.

**Results:**

① There were differences in flora composition and a relative abundance among the groups, but the strains with a high relative abundance were Bacteroides, Firmicutes, and Proteobacteria; ② there were significant differences in the community structure and composition of intestinal flora between nude mice treated for 4 weeks and those not treated (*p* < 0.05); ③ after 4 weeks of administration, the relative abundance of Bacteroidetes in each group was higher than that before administration, and the relative abundance of Firmicutes decreased.

**Conclusion:**

Asini Corii Colla, turtle carapace glue, and other drugs with different compatibility ratios can change the composition of intestinal flora in nude mice with uterine fibroids to a certain extent; the decrease in the relative abundance of Firmicutes and the increase in the relative abundance of Bacteroidetes were important structural changes of intestinal flora in nude mice at 4 weeks after administration.

## 1. Introduction

Uterine fibroids are benign tumors of the uterine smooth muscle tissue, which occur in women of childbearing age at 30–50 years. Over the last few years, the incidence rate has continued to increase incrementally [1]. It typically occurs clinically as abnormal uterine bleeding, pelvic pain, pelvic mass, menorrhagia, pain, etc.; in severe cases, infertility and abortion may occur, which has a serious impact on women's lives and psychology. The specific pathogenesis of uterine fibroids has not been fully defined, but it is generally believed that high levels of estrogen and progesterone can promote the formation and development of uterine fibroids, that is, uterine fibroids are considered sex hormone-dependent tumors [2].

The article "Effect of Ejiao (Asini Corii Colla) and Turtle Carapace Glue on Gut Microbiota in Nude Mice with Uterine Fibroids Based on High-Throughput Sequencing of 16SrRNA Gene" was published in 2022. Journal: Evid Based Complement Alternat Med.

Modern medicine primarily embraces surgery or hormonal treatment. Some studies have shown that the likelihood of recurrence of uterine fibroids after intervention is 38.24% [3]. For patients with no obvious clinical symptoms and small myomas, surgery is not the best treatment, and hormone treatment alone is difficult to achieve a better curative effect. In the context of hormone therapy, adverse effects such as osteoporosis, hypoestrogenemia, amenorrhoea, and myoma may also continue to develop after withdrawal [4]. Compared with western medicine, traditional Chinese medicine has unique advantages such as being less toxic, having few side effects, simple and safe, and a low recurrence rate [5], so more patients tend to choose traditional Chinese medicine for treatment. In recent years, an increasing number of researchers have begun to study the relationship between intestinal microorganisms and the onset of disease. At present, the research on uterine fibroids and intestinal microorganisms is still relatively limited, but some studies have shown that the number and strains of intestinal flora are related to the occurrence of uterine fibroids [6]. Therefore, on the basis of previous experiments, this study conducted biodiversity sequencing through 16SrRNA to observe the structural changes of intestinal flora of the nude mice with uterine fibroids model under the action of donkey-hide gelatin, turtle shell glue, and other traditional Chinese medicines, providing strong evidence for traditional Chinese medicine to regulate the intestinal microecology of nude mice with uterine fibroids.

## 2. Material

### 2.1. Experimental Animal

25 healthy nude mice, weighing 220 ± 20 g and aged 2-3 months were used in this study.

### 2.2. Experimental Drugs

Experimental drugs were as follows: Ejiao (batch No. 1607040, Dong'e Ejiao Co., Ltd.), turtle carapace glue (batch No. 20180301, Henan Furentang Pharmaceutical Co., Ltd.), *Salvia miltiorrhiza* (batch No. 200401-1, Zhejiang Huisong Pharmaceutical Co., Ltd.), and normal saline.

### 2.3. Main Instruments and Reagents

#### 2.3.1. Instruments

Microplate reader (BioTek, FLx800), TruSeq Nano DNA LT Library Prep Kit (Illumina company), Agilent High Sensitivity DNA Kit, Quant-iT PicoGreen dsDNA Assay Kit, and MiSeq Sequencer were used in this study.

The article "Effect of Ejiao (Asini Corii Colla) and Turtle Carapace Glue on Gut Microbiota in Nude Mice with Uterine Fibroids Based on High-Throughput Sequencing of 16SrRNA Gene" was published in 2022. Journal: Evid Based Complement Alternat Med.

#### 2.3.2. Reagents

1.2% agarose gel, 2% agarose gel, 0.8 times magnetic beads washing liquid (Vazyme VAHTS DNA Clean Beads), 80% ethanol, elution Buffer, and MiSeq Reagent Kit V3 (600 cycles) were used in this study.

## 3. Method

### 3.1. Animal Grouping

25 nude mice that have been modeled (2.2 modeling method) were randomly divided into blank control group (group A), turtle carapace glue administration group (group B), turtle carapace glue and ejiao 4 : 1 mixed group (group C), turtle carapace glue and ejiao 1 : 1 mixed group (group D), and turtle carapace glue and *Salvia miltiorrhiza* (danshen) 1 : 1 mixed group (group E), with 5 mice in each group. A0 represents before administration, A2 represents two weeks after administration, A4 represents four weeks after administration, and the remaining groups are the same as above.

### 3.2. Modeling Method

ELT3 cells were subcultured in RPMI1640 medium containing 10% fetal bovine serum at 37.5°C and a 5% CO_2_ incubator, and a large number of cells were amplified. After passage to a sufficient number, the cells were digested with 0.25% trypsin to make single-cell suspension. A small amount of cell suspension was taken and counted with trypan blue. The living cells account for more than 95%. The cells were treated with ice bath PBS at 1000 rpm × 5 min. After rinsing twice, it was made into 5 × 10^7^ cells/ml cell suspension. The cell suspension was injected subcutaneously into the back of nude mice, and each nude mouse was inoculated subcutaneously with 1 point, no point of 0.2 ml. Including 1 × 10^7^ cells until the tumor grows to 80–100 mm^3^.

### 3.3. Administration Method

The dose of turtle carapace glue was 0.08 g/20 g (20 g was the weight of each nude mouse). Group B: 0.08 g turtle carapace glue; Group C: 0.08 g turtle carapace glue + 0.02 g ejiao; Group D: 0.08 g turtle carapace glue + 0.08 g ejiao; Group E: 0.08 g turtle carapace glue + 0.08 g *Salvia miltiorrhiza.* The preparation method was as follows: dissolve 18 g ejiao, 57.6 g turtle carapace glue, and 14.4 g *Salvia miltiorrhiza* in 36 ml water respectively, heat in a 50 ml centrifuge tube (the cover of the centrifuge tube is tightened and sealed with sealing film), boil for 30 min, dissolve, and repack. After modeling, the drug was administered by gavage once a day, 0.2 ml once, for 4 weeks, as shown in Table 1.

### 3.4. Microbial Classification and Sequencing Analysis

16SrRNA gene sequencing was performed on the fecal samples of nude mice. The sequencing part is performed by Suzhou Panomic Biomedical Technology Co., Ltd.; the main sequencing process is as follows: (1) DNA extraction: a Nanodrop was used to quantify DNA and the quality of DNA was detected by 1.2% agarose gel electrophoresis. (2) PCR amplification of the target fragment: take the target sequence such as microbial ribosomal RNA or specific gene fragment that can reflect the composition and diversity of flora as the target, design corresponding primers according to the conservative region in the sequence, and add a sample-specific barcode sequence, so as to PCR amplify the variable region of rRNA gene (single or continuous multiple) or specific gene fragment. (3) Purification and recovery of amplification products: 25 *μ*l PCR product was treated by adding 0.8 times the volume of magnetic beads (Vazyme VAHTS DNA Clean Beads). (4) Fluorescence quantification of amplification products: the fluorescent reagent is the Quant-iT PicoGreen dsDNA Assay Kit, and the quantitative instrument is a microplate reader (BioTek, FLx800). According to the fluorescence quantitative results and the sequencing requirements of each sample, each sample is mixed according to the corresponding proportion. (5) Preparation of sequencing library: the TruSeq Nano DNA LT Library Prep Kit of the Illumina company was used to prepare the sequencing library. (6) High-throughput sequencing on the computer: the second-generation sequencing method detects the 16SrRNA sequence and analyzes it through software.

The article "Effect of Ejiao (Asini Corii Colla) and Turtle Carapace Glue on Gut Microbiota in Nude Mice with Uterine Fibroids Based on High-Throughput Sequencing of 16SrRNA Gene" was published in 2022. Journal: Evid Based Complement Alternat Med.

## 4. Data Processing

QIIME software and R script ggplot2 package were used to comprehensively analyze and process the sequencing results, such as alpha diversity, beta diversity, and flora taxonomic composition. Alpha diversity analysis used the Kruskal–Wallis rank-sum test and Dunn's test as post hoc tests. In beta diversity analysis, adonis difference analysis was used to calculate the explanatory degree (*R*2) and significance (*p*) of distance matrix variance. *p* < 0.5 indicates that the difference is statistically significant.

## 5. Result

### 5.1. OTU Analysis of Intestinal Flora

By optimizing the samples of each group, the OTU data of each group are obtained. Finally, the flower petal diagram is shown in Figure 1. A total of 11647 OTUs are obtained in each group, of which 243 OTU data are contained in each group.

### 5.2. Alpha Diversity Analysis

Alpha diversity reflects the richness and diversity of microbial communities. The Chao index represents the species richness in the community, and the Simpson index reflects the species diversity in the community. In these five groups, the Chao index and Simpson index before administration were higher than those four weeks after administration. Although there were differences in the alpha diversity index among the groups, the differences were not statistically significant (*p* < 0.05) (Figure 2).

The article "Effect of Ejiao (Asini Corii Colla) and Turtle Carapace Glue on Gut Microbiota in Nude Mice with Uterine Fibroids Based on High-Throughput Sequencing of 16SrRNA Gene" was published in 2022. Journal: Evid Based Complement Alternat Med.

With the continuous increase of effective sequencing quantity, Chao1 and Shannon values gradually tend to be stable, indicating that this sequencing is reasonable and representative. The rank abundance curve can be used to explain species richness and evenness. As shown in Figure 3, with the increase of the rank value, the decreasing trend of richness gradually tends to be stable, indicating that the species richness and evenness in the sample are good.

### 5.3. Beta Diversity Analysis

Beta diversity analysis reflected the similarity of the sample community composition, and PCoA analysis was used to investigate the difference of beta diversity of intestinal flora in nude mice. The results are shown in Figure 4. The farther the distance in the figure, the greater the difference in species composition between the two samples. The nonadministered samples and 2-week-old samples are close in spatial distance, and most of them overlap, indicating that the intestinal flora of the two groups of samples is highly similar in community structure and composition. The nonadministered samples and the 4-week-old samples are far apart in spatial distance and have been completely separated, indicating that there are significant differences in community structure and composition between the two groups (*p* < 0.05). So it shows that the intestinal environment has changed 4 weeks after administration, and after 4 weeks of administration, the similarity of the community structure between groups B and C and the blank control group is relatively close, and the similarity between groups D and E and the blank control group is quite different.

### 5.4. Intestinal Flora Structure of 15 Groups of Subjects

Sequencing of the v3-v4 region of microbial 16SrRNA gene in the feces of model nude mice was carried out. The results are shown in Figure 5. The higher relative abundance is Firmicutes, Bacteroidetes, and Proteobacteria. Further species difference analysis shows that Firmicutes and Bacteroidetes have a higher relative abundance in the study objects, but compared with the blank control group, the relative abundance of Firmicutes after administration was lower, and the abundance of Firmicutes at 4 weeks after administration was lower than that at 2 weeks after administration. In Bacteroidetes, the changing trend of each group is that the relative abundance at 4 weeks after administration is higher than that without administration, but the relative abundance of groups B, C, and E decreases at 2 weeks after administration, while groups A and D always show an upward trend. In Proteobacteria, the changing trend of each group is that the relative abundance after administration is higher than that before administration, but the relative abundance of groups B and E is higher at 2 weeks than that at 4 weeks, and that of the remaining three groups is higher at 4 weeks than that at 2 weeks. When observing the ratio of Firmicutes and Bacteroidetes, it is found that at 2 weeks, the ratios of group B and E is higher than that before administration, while the ratios of the other three groups are lower than that before administration, the ratios of group B2 and E2 were higher than the ratio of group A2, while the ratios of the other three groups were lower than the ratio of group A2; at 4 weeks of administration, the ratios of the five groups after administration were lower than those before administration, and those of B4, C4, D4, and E4 were lower than the ratio of A4.

The article "Effect of Ejiao (Asini Corii Colla) and Turtle Carapace Glue on Gut Microbiota in Nude Mice with Uterine Fibroids Based on High-Throughput Sequencing of 16SrRNA Gene" was published in 2022. Journal: Evid Based Complement Alternat Med.

### 5.5. Cluster Analysis of Species Composition among Samples

The double cluster genus level species composition heat map shows that there is a certain clustering trend among most samples before administration and among most samples after administration, suggesting that there are some differences in species composition between samples before and after administration (Figure 6).

### 5.6. LEfSe Analysis of Different Flora among Different Groups

LEfSe analysis can find biomarkers with statistical differences between groups. Using linear discriminant analysis (LDA) = 2 as the threshold, the characteristic flora of each group was screened. It can be seen from the LEfSe multilevel species hierarchy diagram that there are differences in flora in phyla, class, order, family, and genus between the drug group and the nondrug group. The dominant bacteria in group A0 were *Streptococcus*, *Lactobacillus*, Firmicutes, and so on; the dominant strains in group A2 were *Actinomycetes* and *Bifidobacteria*; The dominant strains in group A4 were desferriobacteria and anaerobic *Cladosporium*; the dominant bacteria in group B2 were TM7, and the dominant bacteria in group B4 were Bacteroides and *Bacteroidaceae*; the dominant bacteria in group C2 were *Pediococcus* and *Corynebacterium faecalis*; the dominant strains of the C4 group were beta *Proteus*, etc.; the dominant strains of the D0 group are soft wall bacteria, *Acinetobacter*, anaerobic plasma, etc.; the dominant strains in group D2 were faecalibacterium prausnitzii and Enterococcaceae; the dominant species in group D4 were *Corynebacterium* and Corynebacteriaceae; the dominant strains of theE0 group are Dipteroides, etc.; the dominant bacteria of group E2 are *Shigella* and Enterobacteriaceae; the dominant strains of group E4 are Bacteroidetes and so on, as shown in Figure 7.

The article "Effect of Ejiao (Asini Corii Colla) and Turtle Carapace Glue on Gut Microbiota in Nude Mice with Uterine Fibroids Based on High-Throughput Sequencing of 16SrRNA Gene" was published in 2022. Journal: Evid Based Complement Alternat Med.

## 6. Discussion

The incidence rate of uterine fibroids in women of childbearing age is as high as 20–40% [7], and shows a genetic tendency. The rate of malignant transformation is in the range of 0.4%–1.25% [8]. The majority of patients have no obvious symptoms. The pathogenesis of uterine fibroids is still unclear, but studies had shown that the occurrence of uterine fibroids is related to cellular factors, bypass effects, growth factors, hormone causes, etc. [9]. At present, western medicine mainly adopts hormone therapy and surgical therapy, with a high rate of recurrence and many adverse reactions, which results in a decrease in the quality of life of patients. In traditional Chinese medicine, “uterine fibroids” are classified into the categories of “symptoms” or “accumulation.” In the early stage, many doctors believed that the occurrence of uterine fibroids was mostly related to the damage of Chong Ren Qi and blood, improper adjustment of menstrual production, weakness of viscera, internal and external pathogens, emotional disorder, improper diet, and so on [10]. Later medical practitioners believe that the key to the pathogenesis of uterine fibroids is internal obstruction of blood stasis, which is understood from a modern medical perspective to mean that the blood flow is “thick,” “sticky,” “clotted,” and “gathered” [11]. The previous experiments of our research group had also proved that donkey-hide gelatin and turtle shell glue might have played an antiuterine fibroid role by improving uterine fibroids, reducing the E2 level, and increasing the FSH and LH level [12]. Modern pharmacological studies had found that the main effective component of the turtle shell glue was a turtle shell polysaccharide [13], which had the effects of antitumor, antivirus, and enhancing immunity [13, 14]. Donkey-hide gelatin also had the effects of anti-inflammatory, regulating hormone level, antitumor, and regulating immune function [15–17]. In addition, Colla Corii Asini, turtle carapace glue, and other traditional Chinese medicines have certain antiuterine fibroids effects, and have broad application prospects in the treatment of gynecological diseases.

The purpose of this study is to analyze the effects of Colla Corii Asini, turtle carapace glue, and other drugs on uterine fibroids from the perspective of modern medicine, and analyze the changes of the intestinal flora structure of uterine fibroids in rats after intervention with Colla Corii Asini, turtle carapace glue, and other drugs by 16SrRNA gene sequencing technology. The results of the alpha diversity analysis showed that the abundance and diversity of intestinal flora showed an upward trend after administration, but there was no significant difference, which may be related to the short research time. The results of beta diversity analysis showed that the flora structure of rats at 4 weeks of administration was significantly different from that before administration, and the flora structure of groups A, B, and C showed a similar trend at 4 weeks of administration, and there were significant differences between groups D and E compared with the other three groups. Species composition analysis showed that after 4 weeks of administration, Firmicutes decreased, Bacteroidetes and Proteobacteria increased, Firmicutes/Bacteroidetes ratio decreased, and from the point of view of the ratio of firmicum/Bacteroides, B4, C4, D4, E4 groups were lower than A4 group. Firmicutes and Bacteroidetes are the two bacteria with the highest abundance in the human intestine [18], and the change of their abundance ratio is a marker for reflecting the intestinal microorganisms of obese people [19]. The proportion of Firmicutes/Bacteroidetes in the intestines of obese people is higher than that of normal-weight people [20], and studies such as [21] show that the number of Bacteroidetes in the intestines of obese people is significantly less than that of nonobese people. Over the past few years, studies have demonstrated a positive correlation between obesity and uterine fibroids. Every 10 kg of weight gain in women can increase the risk of uterine fibroids by 21%, or every 1 unit of the body mass index can increase the risk of uterine fibroids by 6% [22]. Human adipose tissue can convert androgen from the adrenal gland and ovary into estrogen [23]. Uterine fibroids are hormone-dependent tumors, and the increase in estrogen levels considerably increases the risk of uterine fibroids. Zhang Yafang et al. [6] found that the levels of Bacteroides and Proteobacteria in the uterine fibroids group were significantly lower than those in the blank control group, and Bacteroides and Proteobacteria were negatively correlated with the incidence of uterine fibroids. The results of this experiment show that medications in all four treatment groups may reduce the ratio of Firmicutes and Bacteroides. The results show that Asini Corii Colla, turtle carapace glue, and other drugs may reduce the estrogen level by reducing the ratio of Firmicutes and Bacteroides and increasing the relative level of Proteobacteria.

The article "Effect of Ejiao (Asini Corii Colla) and Turtle Carapace Glue on Gut Microbiota in Nude Mice with Uterine Fibroids Based on High-Throughput Sequencing of 16SrRNA Gene" was published in 2022. Journal: Evid Based Complement Alternat Med.

TNF-*α* produced by phagocytes is a major inflammatory factor in organisms. It can promote the release of a variety of inflammatory mediators, strengthen the inflammatory response, and cause the proliferation of damaged smooth muscle cells. TNF-*α* is related to the occurrence of uterine fibroids, which may be due to the inhibition of the immune state of the body [24]. The research of Xie and Li [25] has shown that the Biejiajian pill can significantly inhibit TNF-*α* expression. The Biejiajian pill with turtle shell as its king medicine is one of the first three prescriptions in the synopsis of the golden chamber [26]. At the same time, some studies have shown that the Biejiajian pill can inhibit the expression of TNF-*α* to inhibit the growth of uterine fibroids [27]. Duguanhua [28] found the following at the phylum level: there was a positive correlation between the content of TNF-*α* and Firmicutes, on the contrary, Bacteroidea and the content of TNF-*α* was negatively correlated. In addition, reducing the ratio of Firmicutes to Bacteroides can normalize the intestinal microbial community and restore the damaged intestinal barrier function [29]. Combined with the experimental results, we speculate that Asini Corii Colla and turtle carapace glue may inhibit the expression of TNF-*α* by decreasing the ratio of Firmicutes and Bacteroides, thereby reducing the inflammatory response, and thus exerting a therapeutic effect. In addition, our previous experiments have known that high doses of Asini Corii Colla and turtle carapace glue can reduce the level of estradiol, thus playing a role in the treatment of uterine fibroids [12]. Li et al. [17] found that compound ejiao granules can regulate hormone levels and reduce estradiol levels in adult rats. This experimental result is basically consistent with our previous experimental results. At the same time, some studies have found that the relative abundance of Bacteroidetes is negatively correlated with estradiol [30]. Combined with the results of this experiment, we can speculate that Asini Corii Colla and turtle carapace glue may reduce the level of estradiol by increasing the relative abundance of Bacteroidetes, thus exerting an antiuterine fibroid effect.

There are many similarities between the intestinal flora and the theory of traditional Chinese medicine. The Yellow Emperor's Canon of Internal Medicine says the following: “the healthy Qi is stored in the body, and the evil cannot be done. If the evil is gathered together, the Qi will virtual.” Healthy Qi is the key factor to determine the occurrence of diseases, evil Qi is an important condition for the occurrence of diseases, and the struggle between healthy and evil Qi is the basic principle for the occurrence and development of diseases [31]. Regulating the balance of intestinal flora in modern medicine is the biological basis of the theory of “supporting the right and expelling the evil” in traditional Chinese medicine [32]. Modern microecology shows that the intestinal microecology in the human body is in a relatively balanced state, which is the category of “healthy Qi.” When the human body is affected by some other abnormal factors, the microecological balance will be destroyed and imbalanced, which belongs to the category of “evil Qi” [33]. The intestinal flora in the human body is in balance because of the presence of positive Qi, but when the body is affected in some way and this balance is disturbed, microecological disorders occur and the microecological system in the body is transformed from “positive Qi” to “negative Qi,” and disease occurs [34]. Chinese medicine has a multitarget mechanism of action in the treatment of uterine fibroids, and also has a certain effect on the regulation of intestinal flora, but this experiment did not reveal the specific mechanism of the effect of Chinese medicine on intestinal flora, and the current research on Chinese medicine to improve intestinal flora is still insufficient, and more experiments are needed to prove this in the future. In addition, the study period of this experiment was too short to observe the long-term effects of the drug on intestinal flora, and the experiment was only at the level of animal experiments, lacking supporting clinical data. In future studies, the study period can be appropriately extended, and animal experiments can be combined with clinical studies to provide more sufficient evidence for the clinical use of the drug.

The article "Effect of Ejiao (Asini Corii Colla) and Turtle Carapace Glue on Gut Microbiota in Nude Mice with Uterine Fibroids Based on High-Throughput Sequencing of 16SrRNA Gene" was published in 2022. Journal: Evid Based Complement Alternat Med.

In conclusion, Asini Corii Colla and turtle carapace glue with different compatibility ratios can reduce the relative abundance of Firmicutes and increase the relative abundance of Bacteroidetes, may reduce the levels of estrogen and estradiol and inhibit TNF-*α* by regulating the balance of intestinal flora, and play a certain therapeutic role in uterine fibroids.

## Figures and Tables

**Figure 1:** Petal diagram of the sample (group) ASV/OTU.

**Figure 2:** Grouping box diagram of the alpha diversity index.

**Figure 3:** Abundance grade curve.

**Figure 4:** Two-dimensional ranking diagram of samples for PCoA analysis.

**Figure 5:** Histogram of species composition at the phylum level.

**Figure 6:** Heat map of species composition at the genus level.

**Figure 7:** Histogram of the LDA effect value of marker species.

**Table 1:** Group of nude mice and gavage medicine.

Group	Gavage volume (ml)	Gavage medicine
A	0.2	Normal saline
B	0.2	Turtle carapace glue
C	0.2	Turtle carapace glue and ejiao 4 : 1 mixed
D	0.2	Turtle carapace glue and ejiao 1 : 1 mixed
E	0.2	Turtle carapace glue and danshen 1 : 1 mixed

## Data Availability

The data used to support the findings of this study are available from the corresponding author upon request.
